# Cartoon-Style Image Rendering Transfer Based on Neural Networks

**DOI:** 10.1155/2022/2958338

**Published:** 2022-07-16

**Authors:** Lei Wang

**Affiliations:** College of Arts and Humanities, China University of Mining and Technology, Xuzhou 221116, Jiangsu, China

## Abstract

Cartoon rendering of images is a challenging nonphotorealistic image rendering task, which aims to transform real photos into cartoon-style nonphotorealistic images while preserving the semantic content and texture details of the original photos. Based on the understanding of the characteristics of cartoon images and analysis of the defects of established approaches, this paper improves existing methods. The convolutional neural networks' powerful image processing ability and attention mechanism are utilized to get more fine-grained image features, making the result of rendering more realistic. This paper mainly studies how neural networks can better process cartoon pictures, adjust parameters, and choose training methods. Furthermore, the article proposes a new solution of cartoon-style image rendering based on deep learning. The actual test results of real original images have shown that the model is suitable for cartoon-style image rendering.

## 1. Introduction

Cartoons represent humorous or satirical forms of painting that have a great influence on our lives. Classic cartoon images, such as Mickey Mouse and Donald Duck, have become an irreplaceable part of the post-1990s generation. Disney and Marvel comics are still loved by millions of fans around the world. Animation creates another world that a lot of people yearn for. Reading comics can relax personal mind, improve pupils' imagination, find their own ideas and spiritual sustenance, and see the future belonging to students.

Since computer technology has changed people's daily life, it has significantly impacted on comic creation as well. The research on computer graphics has always been one of the hot fields in the domain of computer science, and its major content includes the representation method of graphics in the computer, the calculation of graphics, and the principle and algorithm of display. In 1962, E. Sutherland from MIT Lincoln Laboratory used the term “Computer Graphics” for the first time in his paper, proving that interactive Computer Graphics is a feasible and useful research field [1, 2]. Thus, Computer Graphics as a new branch of independent science was confirmed. At the beginning of the birth of computer graphics, pioneers were mainly committed to using computer technology to better express the natural world and to truly present the picture seen by bare eyes in the computer system.

At first, scholars used computers to imitate the output of early cameras and gradually began to simulate the reality of images. Computer graphics began to pursue real pictures. With the advancement of technology, the term “Photorealistic Rendering” has been used to describe a range of techniques that mimic the output of cameras [3]. In pursuit of realism, early work studied the process and characteristics of light reflected off surfaces and then explored the equilibrium solution of light reaching various surfaces when reflected in the environment. Overall, realistic rendering is usually based on the scene and the physical model of objects in the scene. It stimulates colors, textures, and other attributes of objects in the scene in order to keep behaviors and characteristics consistent with colors, light, and shadow of nature as far as possible [4, 5]. Therefore, the computer system presents scenes complying with “real” pictures of human cognition. This pursuit of realistic feelings has greatly promoted the development of computer graphics. Realistic rendering technology has been widely used in industrial fields such as CAD and postprocessing of film and television. Meanwhile, it has directly drawn forth the industrial field of “CG rendering” [6].

Rendering technology is widely considered to be inseparable from computer models [7, 8], but in fact, it also includes processing two-dimensional images. If the object is a data type of 2D images, then the corresponding technique is called image space nonphotorealistic rendering, whereas if the object is a data type of 3D model, then the technique is called 3D space nonphotorealistic rendering [9]. According to Gooch's classification theory of nonphotorealistic rendering technology, it can be divided into three categories: simulation of artistic media, interactive generation of users' images, and automatic generation of system images.

First and foremost, with the development of social media networks and the increasing popularity of the gaming market, there is a growing demand for personalized, nonrealistic images. For example, more youngsters tend to post photos or art works with personal features in short video platforms. In online games with social functions, many people also desire to have figures with their own characteristics, which require nonphotorealistic rendering. Furthermore, image processing based on deep learning has been investigated by more scholars, such as super-resolution reconstruction, missing image repair, colorization of black-and-white images, and the extremely popular AI face changing recently. Therefore, this kind of deep learning will definitely affect the blossom of comics.

## 2. Related Studies

In the early stage, nonphotorealistic rendering was primarily used as a supplement to photorealistic rendering [10]. Therefore, nonphotorealistic rendering technology for 3D models has many similarities with photorealistic rendering technology for 3D models in terms of implementation methods [11]. Nonphotorealistic rendering techniques for cartoon-style 3D object space are also rare. Nonphotorealistic rendering is generally defined as a technique that uses computers to simulate the rendering styles of various visual arts [12]. There are great differences between nonphotorealistic rendering and photorealistic rendering in the definition, purposes, and common methods. From the angle of specific rendering methods, photorealistic rendering mainly adopts the way of simulation, while nonphotorealistic rendering usually carries out the stylized process of the material. From the perspective of characteristics, realistic rendering results in the representation of the objective world, while nonrealistic rendering contains subjective expressions. From the point of the effect of the rendering works, realistic rendering will effectively reflect the real physical process, while works of nonrealistic rendering emphasize audiences' emotional cognition rather than visual correctness and usually attach some artistic processing closer to the art works in vision.

With the rapid development of computing technology, more and more researchers have devoted themselves to the study of nonphotorealistic cartoon-rendering algorithms. Lander et al. [13] focused on the relationship between textures and cartoon styles in images and proposed a method to realize cartoon coloring through texture mapping. Claes et al. [14] introduced a fast method to achieve cartoon-style rendering in their paper and smoothed the boundaries in the image during rendering. Cartoon rendering methods based on traditional image processing technology are generally nonparametric methods. Rosa [15] proposed an edge fusion method, which first converts images from RGB color space to Lab color space and performs gradient filtering on the *L* channel alone to obtain maps based on the edge gradient of images. At the same time, the *L* channel is smoothed by grayscale quantization in Lab space. Finally, the edge gradient image is fused with a smoothed image in RGB space, and the resulting image has smooth color blocks and prominent edges, with some characteristics of cartoon style.

Raskar et al. [16] offered a method using image depth and edge information in 2004, which takes advantage of multiple flashlights to shoot images to capture geometric information in the images. This approach separates textures from the image to help nonphotorealistic rendering. Winnemoller et al. [17] in 2006 tried to extract the contour of the image by using the bilateral filter combined with Gaussian difference filter, so as to render the image contour. Yan [18] designed a 2D cartoon-style-rendering algorithm based on scan lines in 2009, which can automatically complete cartoon-style rendering in real time. These methods dealing with traditional image processing technology can only process images with simple texture content and uncomplicated background, because they rely on image filtering and edge detection. Their effect is greatly affected by image content while the generalization ability is poor.

Gatys et al. embraced a texture model based on feature space of convolutional neural networks [19]. In this model, textures would be re-presented according to the relationship between feature maps in each layer of the network. When the object information is made clearer, texture extraction will also capture more content features of natural images [20]. Images are input to neural networks, and then, texture analysis is obtained through feature extraction of different convolutional layers and Gram matrix calculation. Next, the image white noise is input to calculate the loss function of textures in different layers to carry out texture synthesis. The document uses the first method of texture synthesis in the paper to transfer image style of oil painting style. The author uses the middle layer of neural networks for the reconstruction of the content, leaving the maximum pixel values of texture image fusion. Finally, it can get the final image containing different artistic styles of oil painting [21].

From the point of endless work in image processing in recent years, people have more research works and ideas in image processing. New breakthroughs have been made in image stylization, image recognition, video stylization, and other aspects [22, 23]. Researchers will introduce image generation and rendering image editing based on the deep learning into the cartoon style and make use of learning ability of deep neural networks to study the mapping relationship between natural images and cartoon-style images. Image transfer networks based on the deep learning can be used for 2D image style of cartoon rendering tasks, and other methods used for image conversion can also be used for cartoon-style rendering. The former regards cartoon style as a kind of abstract artistic style, while the latter models cartoon-style rendering task as a domain-to-domain conversion task between domain of natural images and domain of cartoon-style images [24].

The existing nonrealistic rendering methods of cartoon style can draw cartoon-style pictures in specific scenes, but they cannot meet the changeable practical application scenes. An excellent cartoon-style nonrealistic rendering algorithm should be able to render natural images with any resolution or any object into a cartoon-style image while keeping the semantic content of the image as far as possible. Nowadays, people's living standard is getting better, and their pursuit of art is also becoming higher. Image stylization algorithm based on deep learning has become more worthy of exploration. In the future, there is a high possibility for deep learning and other related algorithms to achieve results of excellent image stylization. We combine convolutional neural network and attention mechanism to obtain a preliminary improved network and establish the matching and migration algorithm to extract the rendered image features in many aspects.

## 3. Convolutional Neural Network Image Rendering

### 3.1. Convolutional Neural Network

The traditional architecture of convolutional neural networks cannot process high-dimensional image input, and the number of neurons in each layer will increase with the square order of image size [25]. Second, the fully connected multilayer network structure does not take into account the spatial information in the image data, so convolutional neural networks are more suitable for processing image data. CNN is a kind of feed-forward neural network, which is stacked by hierarchical structures composed of multiple groups of convolution computation, activation operation, and downsampling. It is one of the most important algorithms for image processing in deep learning consisting of convolution layers and pooling layers. Furthermore, CNN seeks to extract local features, such as emotional word sequences, by limiting the acceptance domain of implicit layers to a local one. The most important advantage of convolutional neural networks is that they have a significant ability of representation learning with a small number of parameters and convenient training. They can automatically learn feature extraction modules for various tasks in a data-driven way. The feature graph extracted by convolutional neural networks has invariability of translation, which is the biggest reason why convolutional neural networks are suitable for processing image data.

The structure of convolutional neural networks is a simulation of the human visual nervous system. Convolutional layers of convolutional neural networks adopt sparse connection and weight sharing strategy, which greatly reduce the number of learnable parameters in each layer of networks, enabling them to train and predict data efficiently. At the same time, the small number of parameters can greatly reduce the risk of network overfitting. Sparse connection and weight sharing strategy are important reasons for the wide application of convolutional neural networks. At first, one-dimensional convolution was the most widely used type. In one-dimensional convolution layers, the convolution vector matrix is calculated through the width *q* of N filters and the convolution kernel. The weight matrix of filter Fn was expressed as *w* ∈ *R*^*q*  *d*^ to construct local features.

(1) $$\begin{array}{c} c^{n}=f\left(w^{n}⊗X+b^{n}\right). \end{array}$$

Here, ⊗ represents the convolutional operation of the vector*, b* is the bias unit*, d* is the dimension of the word vector, *X* is the feature extracted by the filter, and *f* represents nonlinear activation. The most outstanding ability of convolutional neural networks is their ability of feature extraction, which can adapt to learn feature extractors suitable for different tasks according to data and optimization objectives. Therefore, it has been widely used in various image-processing tasks.

Residual Net was proposed by Kaiming from the Microsoft Research Institute [26]. The structure of ResNet can pass down all the previous parameters and greatly improve the accuracy of the network. When it increases the number of network layers to 50, 101, and 152, good results are obtained, but when the network layers are increased to 1202, the results decrease. Because so many network layers are too thick, it will lead to overfitting. The core of Residual Net is to directly transfer each layer of information to the output, which will not cause degradation with the increase of network layers. On the basis of the increasing network layers, the accuracy rate can also be improved to a certain extent to ensure the integrity of extracted features.

With the proposal of further study of VGG network, VGG16 is still used in many problems of image feature extraction. The network uses 3*∗*3 small convolution kernel for feature extraction and 2*∗*2 maximum pooling layer for debasing dimension. The most commonly used ones are VGG16 and VGG19. The network can be roughly divided into five blocks, each of which consists of several convolutional layers in series, followed by a maximum pooling layer, and the last three blocks are fully connected with layers and softmax classifier. The network of VGG is mainly applied in image feature extraction, with 3*∗*3 filters and 2*∗*2 pooling layer. You can improve performance of the network by deepening it. However, the disadvantage of the network is that there are too many parameters needing more storage space accordingly.

### 3.2. CNN Image Processing

As convolutional neural networks produced good results in image recognition and classification, Gatys et al. applied CNN to the learning of artistic style features, extracted styles based on oil paintings, and combined textures of artistic images with real images, which ultimately obtained artistic painting results with photo content. In the feature extraction process of the style graph, a white noise image is also used, and the Gram matrix of the target image and the style image is calculated for feature matching. The convolution loss of each layer of the two images can be expressed as follows:

(2) $$\begin{array}{c} E_{n}=\frac{1}{4\left(N_{n}^{2}M_{n}^{2}\right)}{\sum_{i,j}\left(G_{ij}^{n}-A_{ij}^{n}\right)}^{2}, \end{array}$$

where *E* represents the image loss result, *A* and *G* represent the feature output in layer *n*, and *N* and *M* represent the filter. The overall style loss function can be expressed as follows:

(3) $$\begin{array}{c} L_{s}\left(a,x\right)=\sum_{i=0}^{n}E_{n}W_{n}, \end{array}$$

where *a* stands for style image, *x* represents the final generated image, and *W* is the weight of the NTH layer loss in the overall loss. Convolutional neural networks use stochastic gradient descent to compare the input content image and style image with the target image. The output result graph is constantly modified through training, and the process is cycled by the gradient descent method. At this time, the derivative of the above formula is obtained:

(4) $$\begin{array}{c} \frac{\partial E_{n}}{\partial F_{ij}^{n}}=\frac{1}{N_{n}^{2}M_{n}^{2}}{\left(G^{n}-A^{n}\right)}_{ij}F^{n}. \end{array}$$

In general, the graph output *F* of layer *n* is more than 0. If *F* is less than 0, the derivative is 0. In order to obtain the characteristic content image with the style image, a white noise image is given. Meanwhile, the style loss and content loss are defined as the total loss function, and the calculation formula is shown as follows:

(5) $$\begin{array}{c} L\left(p,a,x\right)=\alpha L\left(p,x\right)+\beta L\left(a,x\right). \end{array}$$

Here, *α* and *β* are, respectively, the weight ratio of the content and the style of the target image. The result of the loss function is the difference between the final result image and the content and style image. It can be concluded that the loss function gradually decreases with an increasing number of iterations. When the loss function decreases to a stable value, the output target image can be regarded as the result of style transfer. Attention is used to screen out a small amount of important information from a large amount of information and focus on this important information, ignoring most of the unimportant information. The larger the weight is, the more it focuses on its corresponding value, that is, the weight represents the importance of information, and value is its corresponding information. Therefore, we skillfully use the attention mechanism to better obtain the image features and reuse these features in the rendering image, so that the final result is more consistent with the characteristics of human painting.

The strength of CNN lies in that its multilayer structure can automatically learn features, even features of multiple levels. The shallow convolution layer has a small perception domain and can learn features of some local regions, but the deeper layer has a larger perceptual domain and can learn more abstract features. These abstract features are less sensitive to the size, position, and orientation of objects, conducive to improve recognition performance. As Figure 1 shows, the right side is clearly a collection of pixels from many regions. In other words, the image on the left is segmented and the image on the right is aggregated according to different regions. In fact, the network is segmented by features and combined by recognition, and there may be many slow changing processes in the process, as shown in Figure 2.

### 3.3. Optimization of the Network

After the convolution operation, the pooling layer calculates local statistics to extract the most important features. This process allows the pooling layer to reduce the feature dimension, so as to reduce the calculation time and cost of CNN and prevent overfitting problems of the model. There are two common pooling methods: average pooling and maximum pooling. Average pooling is to only average feature points in the neighborhood. Maximum pooling means maximization of feature points in the neighborhood. The operation of pooling is very similar to convolution but different in the algorithm. The calculation of pooling operation is shown in formula (6). In the process of pooling, the internal values are not considered and only the size of the filter is concerned. In average pooling, images correspond to the position of the filter size and then average pixels that are not 0. This method is more sensitive to the characteristics of the background information and reduces errors of the estimator variance increases. Maximum pooling is the location of the corresponding filter on the image size, applying to a maximum of pixels. This method can get more outstanding characteristics of textures and clearer boundaries:

(6) $$\begin{array}{c} h_{m}=\frac{1}{\left|N_{m}\right|}\sum_{i\in N_{m}}\alpha_{i},\\ h_{m,j}=\underset{i\in N_{m}}{\max\alpha_{i,j}}. \end{array}$$

As a result of maximum pooling, the edges are more prominent and the lines are more obvious, and the blurred things in the background will be ignored, making the transfer of styles in the background not obvious. The evenly pooled image is smoother, and the background can transfer features of the original style image without blurring out the details. After the analysis of the cartoon image, the cartoon image often has prominent lines and the background does not need too much color block performance; therefore, this essay chooses maximum pooling in the style transfer of the cartoon image.

Gradient descent is often used in machine learning and artificial intelligence to make the model approximate to the minimum deviation. It is an optimization algorithm. Different optimization algorithms will affect the degree of model convergence and time of model training, so it is very important to choose the most appropriate optimization algorithm. The classical gradient descent method is shown in formula (7). The average loss of all training data is adopted to approximate the objective function:

(7) $$\begin{array}{c} L\left(\theta \right)=\frac{1}{M}\sum_{i=1}^{M}L\left(f\left(x_{i},\theta \right),y_{i}\right). \end{array}$$

For the small-batch gradient descent method, parameters are updated according to different blocks, which reduce the randomness of the descent. Since it is carried out in batches, the overall calculation amount will also be reduced and the speed will be accelerated. When parameters are updated, it is often difficult to choose the learning rate; thus, it is necessary to find a balance between accuracy and speed during setting the learning rate. When the learning rate is high, the speed will improve, but it will affect the accuracy. When the learning rate is low, the speed will decrease while the accuracy improves. When the second-order momentum appears, an optimization algorithm of the adaptive learning rate is generated. At the beginning of the training, a high learning rate is selected to speed up the training. After a period of time, when the model gradient descent reaches a certain degree, the learning rate can be reduced to increase the accuracy. Adam combines the first-order momentum with the second-order momentum and accordingly changes the learning rate of different stages by using their estimation of gradient. The learning rate of each stage has a fixed range, and the parameters are relatively stable.

## 4. Image Style Transfer

### 4.1. Convolution Image Matching

Rendering that used to mimic the appearance of the light now mimics actual behaviors of the light to make the graphics look more realistic; therefore, style rendering is all about matching relationships. For real-time style transfer based on block matching, iterative algorithm, and forward network can be used without training any model. The substitution of style block and content block can be adapted to parallel calculation. Two convolution layers, one two-dimensional convolution layer and one two-dimensional transpose convolution layer, are used at the same time. Through the average maximum value of channel direction, the convolution layer finally calculates the position of the corresponding replacement style block of each block in the content graph.

The extraction size of two-dimensional convolution is 3*∗*3, the step size is 1, and the normalized cross correlation is calculated. When calculating the average maximum value in the channel direction, the 2-d transpose convolution reconstructs the full activation by placing each patch of the best matching style at its corresponding spatial position. We use the attention mechanism to better find the best match, so that each color is included in the final rendering. The design is shown in Figure 3.

### 4.2. Adaptive Image Transfer

It can be seen from the result analysis of the traditional matching real-time style transfer, although the model does not need any training and its speed is greatly improved, it loses a lot of style textures and boundary line information [27]. The result is more like the fusion of two images. From the perspective of adaptive algorithm, ResNet is composed of many Residual Blocks and the basic component of each block is the Residual Unit, which is the combined operation of two convolution layers and skip-connection. Based on ResNet-101 architecture, an early cutoff is attempted in the feed-forward calculation of each Residual Block to reduce the redundancy of the model and save consumption of operation, which can support any style conversion. There is a conversion network and loss function calculation network. The generation of style image is faster than the real-time style transfer based on the block matching method.

The main parts of networks are divided into adaptive normalized transformation network and loss function network [28]. The network calculating the loss function will calculate the loss function of the content graph and the style graph during training. The style transformation network consists of three parts: encoding, adaptive normalization, and decoding. VGG network is used for coding, and the fourth convolutional layer is used to extract the features of content graph and style graph. Ada IN layer can normalize the input content graph. Here, it still makes use of the mean and variance of feature graph calculated by each channel matching content graph and style graph. Adaptive Instance Normalization is an improved algorithm based on Conditional Instance Normalization. In the feature space, the algorithm calculates the mean and variance of each channel of the input content image and style image and matches the normalized results. The reconstruction of content images in this paper is also selected from the fourth layer of VGG network. The feature expression based on this algorithm is shown in the following formula:

(8) $$\begin{array}{c} \text{add}IN\left(x,y\right)=\sigma \left(y\right)\left(\frac{x-u\left(x\right)}{\sigma \left(x\right)}\right)+u\left(y\right). \end{array}$$

## 5. Experimental Results and Analysis

In order to verify the authenticity of the model, all the tested pictures in this essay are actually taken or created. Several groups of images have large differences in styles, mainly to verify the processing effect of the model for different styles of images and also to facilitate the adjustment of model parameters. The training data are mainly used in Microsoft Coco database and the standard black-and-white cartoon database for comparison [29]. The Coco data set mainly includes more than 80,000 real images, while the cartoon database primarily contains more than 1,000 black-and-white cartoon images. In the experiment, the size of each training image is adjusted to 256×256, the batch size is set to 5, and the iteration is 50 thousand times. About two cycles are given on Microsoft Coco training data, and about 160 cycles are given on the cartoon data set. It also uses Adam with a learning rate of 3000–3500.

### 5.1. Basic Image Matching

We need to verify the overall fluency of the model through basic image tests. The style transfer speed of block matching is slower than the speed of the general fast style transfer network. Also, most of the time is spent on the calculation of feature transformation, which accounts for 96% of the total calculation. Its core advantage over the general style transfer is to support images of any style. First, we should ensure that each large area has a corresponding rendering result, as shown in the figure. When the input style image resolution is higher, the conversion time will increase as the image increases, as shown in Figure 4. No matter what the final rendering is, there is some value to be created for the artwork, but the overall layout should not be completely changed.

As shown in Figure 5, the relationship between areas and lines can be clearly seen in Figure D. The boundary of the traditional iterative algorithm is not obvious. At the same time, the final image is more like the fusion of two images, rather than the transfer of styles, and the sense of lines between regions is pretty diluted. For illustration, the traditional method of drawing the body movements of the characters cannot have a perfect style. Although deep learning has solved the referred problems through training, it can also be said that the final rendering result in the figure is relatively stiff. Its content expressions basically prefer to image color segmentation and conversion, and the feeling of emotional style is gradually weakened. With comprehensive consideration, this method has high real-time performance and less loss of style information and boundary information, but lacks expressions of overall artistic emotion.

As shown in Figure 4, CNN-AT indicates that convolutional neural networks use attention mechanism for matching. It is obvious that CNN's two methods take longer time. Because they require more features, the total rendering time is relatively long. However, the rendering results of this network algorithm are more diverse and artistic. Combined with Figure 3, CNN needs to extract and process colors, locations, and other features between American and Chinese objects, which contribute to obtain some potential special information, so as to make the final results diverse.

### 5.2. Adaptive Convolution Transfer Test

Rendering is not only the transfer of color outline but also the detailed description of environment and scenery. These descriptions are described in many ways to highlight the artistic image of a picture. Neural networks are more important to highlight the center and vividly express the connotation of the picture. Therefore, our improved adaptive convolution method is more profound for line extraction and more significant for textures. It has excellent performance in cross style transfer between various types.

As you can see from Figure 6, the lines are clearer. It also displays complex textures, including color textures in complex image areas. The higher the number of convolutional layers is, the better the extraction effect will be; while the lower the number of convolutional layers is, the effect will be like the fusion of two paintings. However, compared with the effect of traditional methods, when more textures exist in high level, there is a lack of style information in low-level extraction. Nevertheless, the background of cartoon image cannot appear too many color blocks and needs to retain the boundary, so it is expected to extract features from low-level convolution. Therefore, this method may create style types that we have not seen before and achieve extremely innovative applications in the practice of comic-style transfer.

## 6. Conclusion

With the rapid advancement of artificial intelligence and machine learning research, it could be assumed that the application of deep learning in the field of artistic creation has profound research values. To sum up, the paper studies experience and knowledge of utilizing neural networks to create art works and discusses the space of art brought by algorithms. It aims to further help other artists to understand neural networks and present art in fantastic ways. Moreover, the comic-style transfer algorithm based on deep learning can generate comic-style images with clear lines, simple backgrounds, and textures. Compared with results of different data sets with different parameters of different methods, this improved algorithm can generate better comic-style transfer effect in particular. Last but not the least, the method referred in this essay has achieved certain effects in the transfer of cartoon style. However, people cannot forget that cartoons in real life have educational significance, even including emotional expressions. Therefore, we need to constantly strive to expand research fields and achieve more details of neural network rendering results in right place.

## Figures and Tables

**Figure 1:** Image area pixel matching.

**Figure 2:** An example of an intermediate process for image rendering.

**Figure 3:** Convolutional image matching schematic diagram.

**Figure 4:** Matching the time scale diagram.

**Figure 5:** Area line matching simulation.

**Figure 6:** Oil painting style rendering simulation.

## Data Availability

The experimental data supporting findings of this study are available from corresponding authors upon request.
